# Hyperspectral Image Classification Model Using Squeeze and Excitation Network with Deep Learning

**DOI:** 10.1155/2022/9430779

**Published:** 2022-08-04

**Authors:** Rajendran T, Prajoona Valsalan, Amutharaj J, Jenifer M, Rinesh S, Charlyn Pushpa Latha G, Anitha T

**Affiliations:** ^1^Makeit Technologies (Center for Industrial Research), Coimbatore, Tamilnadu, India; ^2^College of Engineering, Dhofar University, Salalah, Oman; ^3^RajaRajeswari College of Engineering, Bangalore, Karnataka, India; ^4^School of Engineering and Technology, Kebri Dehar University, Kebri Dehar, Ethiopia; ^5^School of Engineering, Jigjiga University, Jigjiga, Ethiopia; ^6^Saveetha School of Engineering, Saveetha Institute of Medical and Technical Sciences, Chennai, India

## Abstract

In the domain of remote sensing, the classification of hyperspectral image (HSI) has become a popular topic. In general, the complicated features of hyperspectral data cause the precise classification difficult for standard machine learning approaches. Deep learning-based HSI classification has lately received a lot of interest in the field of remote sensing and has shown promising results. As opposed to conventional hand-crafted feature-based classification approaches, deep learning can automatically learn complicated features of HSIs with a greater number of hierarchical layers. Because HSI's data structure is complicated, applying deep learning to it is difficult. The primary objective of this research is to propose a deep feature extraction model for HSI classification. Deep networks can extricate features of spatial and spectral from HSI data simultaneously, which is advantageous for increasing the performances of the proposed system. The squeeze and excitation (SE) network is combined with convolutional neural networks (SE-CNN) in this work to increase its performance in extracting features and classifying HSI. The squeeze and excitation block is designed to improve the representation quality of a CNN. Three benchmark datasets are utilized in the experiment to evaluate the proposed model: Pavia Centre, Pavia University, and Salinas. The proposed model's performance is validated by a performance comparison with current deep transfer learning approaches such as VGG-16, Inception-v3, and ResNet-50. In terms of accuracy on each class of datasets and overall accuracy, the proposed SE-CNN model outperforms the compared models. The proposed model achieved an overall accuracy of 96.05% for Pavia University, 98.94% for Pavia Centre dataset, and 96.33% for Salinas dataset.

## 1. Introduction

With the advancements of remote sensing technology, the use of hyperspectral imaging is becoming increasingly common. The precise classifications of ground features using HSI is a significant research topic that has received a lot of interest. Because of its high resolving powers for good spectra, hyperspectral images have a wide variety of uses in the environmental, medical, defense, and mining. The collection of HSI is dependent on imaging spectrometer deployed in various locations. In the 1980s, the imaging spectrum was created. It was utilized to image electromagnetic waves in the ultraviolet, near-infrared, visible, and midinfrared ranges. The imaging spectrometer can photograph in a variety of continuous and extremely narrow band, allowing every pixel to obtain a completely emitted or reflected spectrum in the wavelength range of interest. As a result, hyperspectral images feature great spectral resolution, multiple bands, and a lot of information. Image corrections, noise reductions, transformations, dimensionality reductions, and classification are the most common methods for processing hyperspectral remote sensing images. As opposed to conventional images, hyperspectral images include a wealth of spectral data. These spectral data could represent the physical structures and chemical structures of the target objects, which supports in classification of image [1].

The purpose of computer remote sensing image classification was to detect and classify data from the environment and surface of Earth on remote sensing image in order for determining the feature data matching to the image data and extricate the valuable feature data. The specific use of automated pattern identification technology in the remote sensing domain is computer classification of remote sensing images. The count of imaging bands in HSI was more than in multispectral image, and the capacity to resolve objects was solid, that is, the higher the spectral resolutions. Thus, because of the higher-dimensional features of HSI, as well as the similarity among the mixed pixels and the spectra, the HSI classification methodology still confronts a number of difficulties; the most significant of those are listed below.

- Hyperspectral image data have a higher dimensionality. Because HSIs are produced by combining values of spectral reflectance acquired by space-borne or airborne imaging spectrometer in hundreds of bands, the related spectrum data dimension of HSIs can likewise be hundreds of dimensions.
- Variability of spectral information in space. The HSIs are affected by atmospheric conditions, structures, and distributions of ground features, sensors, and the surrounding environments.
- The interference of noise and background variables during the capture of hyperspectral images has a significant impact on the quality of the obtained data. The classification accuracy of hyperspectral images is directly affected by the quality of image [1].

Deep neural network's work is based on extracting features from raw input data via processing layer-by-layer of input data. Although the use of spectral characteristics in isolation can be beneficial, it might not be sufficient in many instances. When two diverse items have the similar spectral signatures, their forms and textures can be used to distinguish them. As a result, spectral and spatial data could be merged to enhance HSI classification. Deep networks could extricate spatial and spectral characteristics from HSI data at the same time. However, traditional deep neural networks have significant limitations. They need a large number of training samples and a significant amount of work to tune hyperparameters [2].

Deep learning networks are classified into many types. The convolutional neural networks is one of the most well-known networks for extracting and classifying HSI features [3]. The squeeze and excitation (SE) network was combined with CNN (SE-CNN) in this work to increase its performance in extracting features and classifying HSI images. The squeeze and excitation block is designed to improve the representation quality of a convolutional neural network. In the experiment, three HSI benchmark datasets were utilized for evaluating the proposed model. The proposed model is verified based on the obtained performance by comparing it to the existing approaches used for HSI classification.

## 2. Related Works

Bandar and Munif proposed the deep hypernetwork architecture capable of learning the deep features of HSIs and provided fine performances without the need for dataset augmentation or extensive preprocessing. The primary aim of this HSI classification algorithm was to anticipate the type of land cover by allocating and labelling separate pixels with multiple frequency bands into individual classes. By integrating and merging the basic principles of both Inception and ResNet into a single model, a novel CNN model was presented that used both the deep residual network and inception models. The performance was not improved over conventional techniques because of the minimal volume of labelled training sample [4]. Madhumitha et al. proposed the HSI classification model using an edge detection, optimization, dimensionality reduction, and classification procedures. The image denoising with filter functionality and edge identification method were used to implement the edge detection procedure. The optimization procedure was carried out by first producing the initial populations, then computing fitness, Cauchy mutation, crossover, and lastly determining the decreasing rate with a value of optimal threshold. The input HSI with L-bands was segmented utilizing auto encoder after the denoising was removed, and dimensionality reduction was performed, yielding the output images with *M* components. CNN was used to classify the HSI, and the *M* components were categorized using two stages of convolution and max-pooling. The dimensionality reduction technique in HSI improved overall performance while reducing computing complexity [5].

Xin et al. presented the multisource deep transfer learning framework (MS-DTL). This multisource transfer learning approach was utilized to classify HSIs in order to get more information and ease the problem of limited samples. The ResNet-like basic model was created to address the needs of many sources and a single target. A loss that included the cross-entropy losses from each source HSI was used to train this model. The shallow layers were moved, the number of classes was raised by utilizing various sources to extract global features, and this method's performance was enhanced [6]. Yahya et al. used CNNs to automatically detect haploid and diploid maize seeds using transfer learning-based technique. For this work, AlexNet, VGGNet, GoogLeNet, and ResNet were used particularly. In contrast, the VGG-19 outperformed the others [7]. Fuding et al. proposed a spectral–spatial HSI classification technique based on superpixel pooling CNN and transfer learning (SP–CNN). The model was divided into three phases. The first section comprised of a convolution and pooling operation, which was a down-sampling method used to extract the key spectral features of an HSI. The next section used up-sampling and super-pixel pooling to investigate an HSI's spatial structure information. Finally, the hyperspectral data were loaded into a fully connected neural network using each superpixel as a basic input rather than a pixel [8]. Yakoub et al. proposed a classification of remote sensing scene model based on CNN and other deep transfer learning algorithms. The detailed performance analysis was discussed in [9].

For extracting meaningful features of spectral–spatial from HSI images, Yushi et al. presented the 3-D CNN-based features extraction approach with combined regularization. A regularized deep features extraction technique for HSI classification using CNN was presented. This model extracted deep features from HSIs using multiple convolutional and pooling layers that were discriminant, nonlinear, and invariant. These features were beneficial for classification of image and identification of target. This model has an overfitting problem [10].

Shengjie et al. presented MDL4OW, a multitask deep learning technique for HSI classification with unknown classes, in which a multitask network was used to do classification and reconstruction at the same time. The classification supplied the likelihood of known classes, but the reconstruction estimated the unknown value. According to the findings, the integrity of a classification system was significant in HSI classification with unknown classes [11]. To solve the overfitting problem, Haokui et al. presented AINet, a 3D asymmetric inception network for HSI classification. Initially, AINet utilized a lightweight 3D CNN that was nevertheless highly deep, allowing deep learning to be used to extract representative features and ease the difficulty caused by the restricted annotation datasets. Second, while assessing the HSI's property, spectral signatures were prioritized above geographical contexts. Furthermore, a data fusion transfer learning approach was used to improve model initialization and reduce training time [12].

Xiangyong et al. presented an active deep learning technique for HSI classification that combined active and deep learning into a single framework. First, the CNN was trained with a small quantity of labelled pixels. Following that, the most informative pixels from the candidate pool were actively chosen for labelling. The CNN was then fine-tuned using the newly generated training set, which included the newly labelled pixels. Finally, for improving the classification performance, the Markov random field was used to enforce class label smoothness [13]. From the review of related works, it can be seen that most of the researches used the deep learning techniques for the classification of HSI. Deep learning proved as the best approach for the classification, especially CNN when it comes to image processing. Although, the CNN has some drawbacks of degraded performance due to the overfitting and underfitting issues. To solve these issues, the deep transfer learning techniques can be used, which is a pretrained model that supports to overcome these issues and improves the performance of the model in classification. Different DTL techniques have been proposed earlier, from that the squeeze and excitation network was a recently proposed model that is used in this proposed research with the CNN for the classification of HSI. The SE-Net has an improved performance comparing to the other DTL techniques like Inception, VGG, ResNet, ResNext, and so on.

## 3. Proposed Methodology

The HSI classification model developed in this work is based on a feature extraction method that combines a squeeze and excitation network with a deep convolutional neural network. Deep learning is difficult to apply to HSI because HSI's data structure is complicated. In general, the neural network has a strong representation capability and a larger volume of training samples. The primary objective of this work was to create a deep feature extraction model for HSI classification. Deep networks are capable of extracting spatial and spectral characteristics from HSI data simultaneously, which is advantageous for increasing the performances of the presented model. The SE network was combined with CNN (SE-CNN) in this research to increase its performance in extracting features and classifying HSI.

### 3.1. Convolutional Neural Network

CNN is a feed forward neural network with multiple convolutions and pooling operations, which has the benefits of automated spatial data learning and overfitting issue management. It performs admirably in image recognition, tracking target, and natural language processing. In this work, the CNN method was used for extracting deep HSI classification features. The CNN training method consists mostly of forward propagations and backward parameter updates, and every network layer was described in detail in the following sections.

#### 3.1.1. Forward Propagation Process

CNN convolves input image to the C-layer by using varying widths of the convolution kernel. After applying the bias, the features of abstract textures of the input image were extricated using the activation function to accomplish feature improvement. Convolution could be represented as follows:

(1) $$\begin{array}{c} x_{j}^{l}=f\left(\sum_{i\in M_{j}}x_{i}^{l-1}*w_{ij}^{l}+b_{j}^{l}\right). \end{array}$$

Here, *x*_*i*_^*l*^ was jth factor of lth layer; *M*_*j*_ was jth convolution segment of l-1 layered feature maps; *x*_*i*_^*l*−1^ was the factor in that; *w*_*ij*_^*l*^ was the lth layer's weight matrix; *b*_*j*_^*l*^ was the bias; *f* was commonly the function of nonlinear ReLU activations, and it was represented by,

(2) $$\begin{array}{c} f\left(x\right)=\max\left(0,\;x\right). \end{array}$$

#### 3.1.2. Pooling Layer

The pooling layer, otherwise called as down-sampling layer, was often found beyond the C-layer. It could reduce unnecessary features through employing a down-sampling mechanism for avoiding additional over fitting and parameters of lower networks. Assuming that *l*-1th layer was C-layer, the following *l*th P-layer may be written like,

(3) $$\begin{array}{c} x_{j}^{l}=f\left(\beta_{j}^{l}*down\left(x_{j}^{l-1}\right)+b_{j}^{l}\right), \end{array}$$

where *β*_*j*_^*l*^ indicates the weight and *b*_*j*_^*l*^ indicates the bias of the *l*th layer's *j*th feature map, correspondingly. The down (^*∗*^) symbol represents the function of down-sampling, which usually includes mean, max, and stochastic pooling. To decrease the dimension of output feature maps, the max-pooling with shift-invariances was utilized.

#### 3.1.3. FC Layer

The last FC layer can acquire the output class or the input sample probability after numerous alternative convolution and pooling processes. All neuron nodes in the *k*th layer are linked to every output node in the upper *k*-1th layer in the FC-layer, and its mathematical expression is as follows:

(4) $$\begin{array}{c} y^{k}=f\left(w^{k}x^{k-1}+b^{k}\right), \end{array}$$

where *k* denotes the network layer's numerical order; *y*^*k*^ was the FC-layer outcome; *x*^*k*−1^ was the unfolded single dimension eigen vector; *w*^*k*^ was the weighted coefficient; *b*^*k*^ indicates the bias; and *f* (^*∗*^), activation functions of the last layer in a FC-layer was Softmax functions for classifications operations. Furthermore, after every C-layer or FC-layer, a dropout function called as a regularization approach could be applied to improve the generalization capabilities of proposed CNN approach and minimize overfitting while training the approach [14].

#### 3.1.4. Back Propagation for Parameters Update

The input samples target could be obtained after forward propagation. The network parameters are then returned to their original state by reducing the loss functions of the actual and target outputs. HSI classification may be viewed as an image multiclassification process in this work. As a result, the categorical cross-entropy loss function was used, which can be expressed as:

(5) $$\begin{array}{c} E=\frac{1}{n}\sum_{k=1}^{n}\left[y_{k}\ln\;t_{k}+\left(1-y_{k}\right)\ln\left(1-t_{k}\right)\right], \end{array}$$

where *n* was the sample amount, *y*_*k*_ was the actual target, and *t*_*k*_ was the *k*th sample's predictive value, accordingly. The gradient descent approach could minimize the loss function during model training. The CNN model's adaptive parameters *w* and *b* are gradually updated by computing the partial derivatives of (5). The following are the expressions:

(6) $$\begin{array}{c} w_{ij}^{l}=w_{ij}^{l}-\alpha \frac{\partial E}{\partial w_{ij}^{l}}, \end{array}$$

(7) $$\begin{array}{c} b_{j}^{l}=b_{j}^{l}-\alpha \frac{\partial E}{\partial b_{j}^{l}}. \end{array}$$

In (6) and (7), *α* is the learning rate that controls the parameter updates stride. A suitable *α* may increase network convergence speed and prevent the network from declining into the local optimal solution. As a result, the time-based learning rate schedule used in this study is as follows:

(8) $$\begin{array}{c} \alpha =\alpha *\frac{1}{\left(1+\text{decay}*\text{epoch}\right)}, \end{array}$$

where decay represents the reduction in learning value from the earlier or prior epoch through the particular fixed values; and epoch was present training epoch. At last, the aforementioned back-propagation method completes the whole CNN's training process [15].

### 3.2. Channel Domain Attention

To improve the model's feature extraction performance and therefore to achieve precise classification, the channel attention in Figure 1, SENet, will be used in this work for recalibrating deep featured maps produced by CNNs. SENet could learn global data automatically and apply varying weight ratios for filtering channels to choose target on key features and eliminate unnecessary data using the squeeze and excitation procedures. A series of convolutional transformations F_tr_ can convert the provided image *X*, as input with the dimension of (*W*′, *H*′, *C*′), it could be mapped to the feature map *U* while *U* ∈ *R*^*H *×* W *×* C*^. The output *U* = [*u*_1_, *u*_2_,…, *u*_*C*_] may be written as follows:

(9) $$\begin{array}{c} u_{c}=v_{c}*X=\sum_{s=1}^{C{}^{\prime }}v_{C}^{s}*X^{s}. \end{array}$$

where *∗* represents the convolution operation; *V* =  [*v*_1_, *v*_2_ … *v*_*C*_] denotes the learnt convolution kernels; and *v*_*C*_  =  [*v*_*c*_^1^,  *v*_*C*_^2^ … *v*_*C*_^*c*^] is the *C*th 2D spatial filter kernels; *X* = [*x*^1^, *x*^2^, ..., *x*^*C*′^] and *u*_*c*_ ∈ *R*^*H*×*W*^. The squeeze transform F_sq_ then translates feature mappings *U* to the global spatial single dimension feature vectors, and a statistic z ∈ *R*^*C*^ produced by compacting U with spatial dimension *H *×* W* may be expressed as follows:

(10) $$\begin{array}{c} z_{c}=F_{sq}\left(u_{c}\right)=\frac{1}{H\times W}\sum_{i=1}^{H}\sum_{j=1}^{W}u_{c}\left(i,\;j\right). \end{array}$$

According to (10), the above procedure was a global average pooling for obtaining the statistic *z*. Hence, using the self-gating method with dual FC-layers, the excitation operation was developed for performing evaluation of weight on all channels for adaptive featured recalibrations. It may be written as follows:

(11) $$\begin{array}{c} s=F_{ex}\left(z,\;W\right)=\sigma \left(g\left(z,\;W\right)\right)=\sigma \left(W_{2}\delta \;\left(W_{1},\;z\right)\right). \end{array}$$

where *δ* was the ReLU activation function, *W*_1_ ∈ *R*^*C*/*r*×*C*^ and *W*_2_ ∈ *R*^*C*×*C*/*r*^, and *r* represents a ratio of dimensionality reduction. At last, the SE block's output was obtained by rescaling *U* with the activation *s*.

(12) $$\begin{array}{c} {\tilde{X}}_{c}=F_{\text{scale}}\left(u_{c},\;s_{c}\right)=s_{c}\cdot u_{c}, \end{array}$$

where $\tilde{X}=\left[{\tilde{X}}_{1},\;{\tilde{X}}_{2},\ldots ,\;{\tilde{X}}_{c}\right]$ and *F*_scale_(*u*_*c*_,  *s*_*c*_) signify channel-wise scalar multiplication *s*_*c*_ and feature map *u*_*c*_ ∈ *R*^*H*×*W*^ [17].

The descriptive realization procedure of SE-CNN model was on the basis of theoretical analysis discussed above, where the deep featured maps were extricated initially by a CNN approach, and single dimension weighted vectors of filter channel were acquired by the group of consecutive performances comprising FC-layer, global pooling, ReLU, and Sigmoid activations in Figure 2. Thus, for precise image identification, the feature maps generated by the CNN were recalibrated utilizing the aforementioned channel weight ratio. As a result, this research will integrate CNN and SENet for creating a SE-CNN model for HSI classification.

To train the CNN model more easily, the image size was typically 2^*n*^, such as 32, 64, 128, 256, and so on. In addition, based on the efficiency of detection and HSI classification accuracy, this model resizes the image as 64 × 64 pixels in size. Following that, the SE-CNN model was created for extracting deep features in comparison to other CNN models. For input images, the SE-CNN model has several interchanging P-layers and C-layers, as well as one or few FC-layers.

Each of the aforementioned CNN models has 32, 32, 64, or 128 filters in its C-layer, and strides of P-layers and C-layer performances were fixed to one. In addition, a zero-padding approach with the same padding was used on CNN models for keeping feature maps the same size. The SE module recalibrates the CNNs' output feature maps, including squeeze, excitation, and scale procedures. Finally, the FC-layers flatten the calibrated feature maps, allowing a Softmax classifier to classify the images.  Table 1 represents the particular parameters of the proposed deep learning model, where *C*_1_∼*C*_4_ denotes the convolutional layers, *P*_1_∼*P*_4_ denotes the max-pooling layers, and FC-layer finally for HSI classification. Furthermore, the models described above all were applied with batch normalization following the initial C-layer and trained with a batch size of 32. Simultaneously, to prevent the network from overfitting, a dropout operation was presented after the FC-layer. Because the SE module's dimensionality reduction ratio *r* impacts classification accuracy, relevant tests and analysis are carried out in this research.

## 4. Experiment Analysis

This section focuses on and presents a detailed review of experiments based on HSI classification utilizing three HSI datasets. Two evaluation measures were utilized to assess the proposed method's efficiency in distinguishing different classes of hyperspectral images. The accuracy of all classes in the testing set was determined as the first measure, and the overall accuracy was the second measure, which was computed as the total of properly classified hyperspectral samples split by the overall count of HSI samples in testing set. To demonstrate the validity of the proposed technique, different existing classification methods for hyperspectral imagery were used for the comparison, namely, VGG-16, Inception-v3, and ResNet-50. MATLAB 2017a was used to run the tests using a system with Intel core i5 CPU with 2.9 GHz speed, RAM with 8 GB, and a 64 bit Windows 10-OS [18–25].

### 4.1. Dataset Description

In this research, three HSI benchmark datasets such as Pavia Centre, Pavia University, and Salinas, were utilized for evaluating the proposed approach, and their descriptions are as follows.

#### 4.1.1. Pavia Centre and University Datasets

Pavia Centre and University are two images captured by the ROSIS sensor during the fly above Pavia, Italy. Pavia University has 103 spectral bands, where Pavia Centre has 102. Pavia Centre has the 1096 × 1096 pixels images, while Pavia University has the 610 × 610 pixels images although some samples in both images are insufficient in information and deleted before processing. The spatial resolution was 1.3 meters. Both image ground truths distinguish nine groups.  Table 2 represents the description of the Pavia Centre dataset, and Table 3 represents the description of the Pavia University dataset.

#### 4.1.2. Salinas

This dataset was collected by the airborne visible/infrared imaging spectrometer (AVIRIS) sensor above the city of Salinas Valley, California, USA. This collection incorporates images with the size of 512 × 217 pixels, a spatial resolution of 3.7 meters, and 204 bands after eliminating 20 water absorption bands. The accessible ground references map includes 16 different classes, such as vegetables, vineyards, and bare soil as shown in Table 4.

Figure 3 represents the ground truth images of the datasets utilized in this research for evaluation. It is worth noting that the zero value in the ground truth maps displayed in Figures 3(a)–3(c) indicates clutter pixels, which could not be classified as a new class.

### 4.2. Performance Analysis

For the performance evaluation, the datasets are divided into 50% to train and 50% to test. As shown in the following tabulations, Table 5 represents the accuracy of every class and overall accuracy of total classes based on the classification performance of the proposed model using the Pavia Centre dataset. This Pavia Centre dataset is divided into 3728 samples for training and 3728 samples for testing for the experiment. The classification performance of the proposed model was compared with other existing deep transfer learning approaches like Inception-v3, VGG-16, and ResNet-50.

As shown in Table 5, the proposed model has obtained better classification results in most of the classes and obtained an overall accuracy of 98.94%, which is 1.04–2.01% improved than the other compared models. The Inception-v3 and ResNet-50 models have achieved some best results in few classes compared to the proposed model, and in most classes, both these models achieved some close results.  Figure 4 represents the graphical plot of overall accuracy obtained by the models.

Table 6 represents the evaluation of the classification performances of the proposed model based on the accuracy achieved on every class and the overall accuracy of the proposed model using the Pavia University dataset. The Pavia University dataset is divided into 21388 samples for training and 21388 samples for testing in this performance evaluation. As noted in Table 6, the proposed model has obtained better classification results in majority of classes and obtained an average accuracy of 96.05%, which is 0.48–1.2% improved than the other compared models. The Inception-v3 and ResNet-50 models have achieved some best results in few classes compared to the proposed model, and in most classes, both these models achieved some close results. VGG-16 has the least performance in this evaluation.  Figure 5 represents the graphical plot of accuracy acquired by the models with Pavia University dataset.

Table 7 represents the classifications performance evaluation of the proposed system based on the accuracy obtained in every class and the overall accuracy of the proposed system using the Salinas dataset. Salinas dataset is divided into 27065 samples for training and 27064 samples for testing in this performance evaluation.

The above table shows that the proposed model has obtained better classification results in many classes and obtained an overall accuracy of 96.33%, which is 1.18–5.9% improved than the other compared models. The Inception-v3 and ResNet-50 models have obtained better results in one or two classes than the proposed model. In most classes, both these models obtained some close results. VGG-16 has the least performance in all these experiment evaluations.  Figure 6 represents the graphical plot of accuracy acquired by the models with the Salinas dataset.  Figure 7 represents the graphical plot of accuracy acquired by the proposed model based on the three datasets used in this research.

## 5. Conclusion

In this research, the HSI classification model was proposed based on a feature extraction method that combined a squeeze and excitation network with a deep convolutional neural network. The primary objective of this research was to create a deep feature extraction model for HSI classification. Deep networks were capable of extracting spatial and spectral features from HSI data simultaneously, which is a benefit for enhancing the performance of the proposed model. The squeeze and excitation network was proposed in this work for this feature extraction model utilizing CNN. The squeeze and excitation block was designed to improve the representation quality of a convolutional neural network. Three benchmark datasets, such as Pavia Centre, Pavia University, and Salinas, were utilized in the experiment to evaluate the proposed model. The proposed model's performance was validated by a performance comparison with current deep transfer learning approaches such as Inception-v3, VGG-16, and ResNet-50. The proposed SE-CNN model outperforms the compared models in terms of accuracy across all dataset classes as well as overall accuracy. The proposed model achieved an overall accuracy of 98.94% for Pavia Centre dataset, 96.05% for Pavia University dataset, and 96.33% for the Salinas dataset. The time required to train the proposed model is the primary drawback of this study. In future, this limitation will be solved by improving the preprocessing function and adjusting the number of layers in the network and finding a solution for solving the data imbalance in HSI classification.

## Figures and Tables

**Figure 1:** Squeeze and excitation block [16].

**Figure 2:** Proposed SE-CNN model for HSI classification.

**Figure 3:** Ground Truth images: (a) Pavia University; (b) Pavia Centre; (c) Salinas.

**Figure 4:** Graphical plot of overall accuracy on Pavia Centre dataset.

**Figure 5:** Graphical plot of overall accuracy on Pavia University dataset.

**Figure 6:** Graphical plot of overall accuracy on Salinas dataset.

**Figure 7:** Proposed model's accuracy on each dataset.

**Table 1:** Parameters of CNN model.

Layer	Parameters
Input	Input image with a size of (64 × 64, 3)
C_1_	Conv 2D (32, 3 × 3)
BN_1_	Batch normalization
P_1_	Maxpooling 2D (2, 2)
C_2_	Conv 2D (32, 3 × 3)
P_2_	Maxpooling 2D (2, 2)
C_3_	Conv 2D (64, 3 × 3) drop out (0.35) ReLU
P_3_	Maxpooling 2D (2, 2)
C_4_	Conv 2D (128, 3 × 3)
P_4_	Maxpooling 2D (2, 2)
FC_1_	1024
FC_2_	256
Output	Classification of images

**Table 2:** Pavia Centre dataset description.

Class	Sample
Water	824
Trees	820
Asphalt	816
Self-blocking bricks	808
Bitumen	808
Tiles	1260
Shadows	476
Meadows	824
Bare soil	820
Total	7456

**Table 3:** Pavia University dataset description.

Class	Sample
Asphalt	6631
Meadows	18649
Gravel	2099
Trees	3064
Painted metal sheets	1345
Bare soil	5029
Bitumen	1330
Self-blocking bricks	3682
Shadows	947
Total	42776

**Table 4:** Salinas scene dataset description.

Class	Sample
Corn_senesced_green_weeds	3278
Celery	3579
Brocoli_green_weeds_1	2009
Fallow_smooth	2678
Fallow	1976
Brocoli_green_weeds_2	3726
Fallow_rough_plow	1394
Soil_vineyard_develop	6203
Stubble	3959
Vineyard_untrained	7268
Grapes_untrained	11271
Lettuce_romaine_6 wk	916
Lettuce_romaine_4 wk	1068
Vineyard_vertical_trellis	1807
Lettuce_romaine_7 wk	1070
Lettuce_romaine_5 wk	1927
Total	54129

**Table 5:** Evaluation of accuracy on each class of Pavia Centre dataset with overall accuracy.

Class	VGG-16	Inception-v3	ResNet-50	Proposed
Water	99.89	100	100	100
Trees	94.85	95.78	95.10	95.43
Asphalt	93.90	96.39	96.02	95.18
Self-blocking bricks	87.56	89.08	90.17	90.38
Bitumen	95.44	96.71	96.50	97.84
Tiles	96.34	98.58	98.49	98.95
Shadows	95.04	95.20	94.99	95.46
Meadows	97.63	98.05	98.57	99.65
Bare soil	96.50	96.89	98.17	99.68
Overall accuracy	96.93	97.90	97.55	98.94

**Table 6:** Evaluation of accuracy on each class of Pavia University dataset with overall accuracy.

Class	VGG-16	Inception-v3	ResNet-50	Proposed
Asphalt	93.85	92.61	96.20	96.89
Meadows	96.04	96.35	97.52	98.74
Gravel	78.33	81.26	80.09	81.63
Trees	90.12	96.79	96.62	96.08
Painted metal sheets	99.90	100	99.85	100
Bare soil	89.44	91.73	94.26	93.38
Bitumen	85.60	90.83	86.90	89.16
Self-blocking bricks	86.75	89.48	92.07	92.94
Shadows	100	99.73	99.97	100
Overall accuracy	94.85	95.14	95.57	96.05

**Table 7:** Evaluation of accuracy on each class of Salinas dataset with overall accuracy.

Class	VGG-16	Inception-v3	ResNet-50	Proposed
Brocoli_green_weeds_1	98.74	99.56	99.38	99.65
Brocoli_green_weeds_2	97.49	99.89	99.60	99.96
Fallow	98.50	99.93	100	99.92
Fallow_rough_plow	98.87	99.50	99.10	99.44
Fallow_smooth	98.79	98.27	99.74	99.50
Stubble	96.00	96.80	99.28	99.81
Celery	98.94	99.13	99.41	99.90
Grapes_untrained	86.52	91.95	93.82	94.14
Soil_vinyard_develop	99.87	100	100	100
Corn_senesced_green_weeds	94.38	97.58	98.25	97.40
Lettuce_romaine_4 wk	93.82	97.75	99.01	98.57
Lettuce_romaine_5 wk	97.06	99.49	99.72	99.80
Lettuce_romaine_6 wk	98.31	99.24	98.90	99.35
Lettuce_romaine_7 wk	91.95	98.89	99.05	99.26
Vinyard_untrained	65.15	78.36	81.29	82.90
Vinyard_vertical_trellis	97.87	98.21	99.00	99.28
Overall accuracy	90.43	92.89	95.15	96.33

## Data Availability

The datasets used and/or analyzed during the current study are available from the corresponding author on reasonable request.
